# A novel methylation signature predicts inferior outcome of patients with PDAC

**DOI:** 10.18632/aging.202347

**Published:** 2021-01-10

**Authors:** Minqi Gu, Jing Sun, Shunhao Zhang, Jing Chen, Guihua Wang, Shaoqing Ju, Xudong Wang

**Affiliations:** 1 Department of Laboratory Medicine, Affiliated Hospital of Nantong University, Nantong, Jiangsu, China; 2 School of Public Health, Nantong University, Nantong, Jiangsu, China

**Keywords:** DNA methylation, pancreatic ductal adenocarcinoma, The Cancer Genome Atlas, prognosis

## Abstract

Pancreatic ductal adenocarcinoma (PDAC) will become the second most common cause of death in North America and Europe over the next 10 years owing to the lack of early diagnosis, poor treatment, and poor prognosis. This study evaluated the methylation array data of 184 patients with PDAC in The Cancer Genome Atlas database to explore methylation biomarkers related to patient outcome. Using Univariable Cox regression analysis and Lasso regression analysis method in the training dataset, it was found that the four DNA methylation markers (*CCNT1*, *ITGB3*, *SDS*, and *HMOX2*) were significantly correlated with the overall survival of patients with PDAC. Kaplan–Meier analysis showed that these four DNA methylation markers could significantly distinguish high-risk and low-risk patients. Receiver operating characteristic analysis further confirmed that the four DNA methylation markers had high sensitivity and specificity, which could predict the prognosis of patients. Moreover, there was a difference in the genetic mutations between high-risk and low-risk patients distinguished by the four-DNA methylation model, which can provide information for clinical treatment. Finally, compared with known biomarkers, the model was more accurate in predicting the prognosis of PDAC. This four-DNA methylation model has potential as a new independent prognostic indicator, and could be used for the diagnosis, monitoring, and precision medicine of pancreatic cancer.

## INTRODUCTION

Pancreatic cancer is an insidious and rapidly progressing digestive system neoplasm. It ranks second among the causes of digestive system cancer-related death [1]. Pancreatic ductal adenocarcinoma (PDAC) is the most common pathological type, and accounts for 90% pancreatic cancers [2]. Owing to the deep anatomical location of the pancreas and the lack of specific markers of PDAC, most patients are diagnosed at the advanced tumor stage [3, 4]. Currently, surgical resection is the most effective method for PDAC treatment. With the rapid development of medicine, several targeted drugs have been developed for clinical practice [5, 6]. However, postoperative patients with PDAC often frequently relapse and have poor prognosis because of micro-infiltration and micro-metastasis in the lesions. The 5-year survival rate of PDAC is only 1%–3% [7]. Therefore, to improve the clinical outcome of PDAC, identifying novel biomarkers that can stratify the risk of patients and predict their survival time is valuable for guiding therapy for PDAC. In this study, patients with PDAC were divided into high-risk and low-risk groups according to the risk index. These two groups could undergo different strategies to reduce the side effects caused by same therapeutic regimen. The establishment of a specific model that identifies high-risk patients is urgent for clinical management of PDAC.

DNA methylation is an important epigenetic modification, during which a specific base of a DNA sequence catalyzed by methyltransferase and s-adenosylmethionine is used as a methyl donor to obtain a methyl group by covalent bonding. [8]. The cytosine of the dinucleotide CG (CpG sites) is a common site of DNA methylation, and these genomic regions rich in CpG sites are called CpG islands [9]. It is well known that DNA methylation can change chromatin structure, DNA conformation, DNA stability, and the interaction between DNA and proteins to regulate gene expression. There are two main forms of DNA methylation regulation gene expression, namely high methylation of tumor suppressor genes and low methylation of oncogenes. High methylation of tumor suppressor genes can significantly inhibit the expression of genes and prevent them from exerting their ability to suppress tumors. Effect, leading to unlimited growth of tumors; hypomethylation of oncogenes can activate oncogenes and promote tumor growth. Aberrant DNA hypomethylation is one of the main abnormalities of tumor DNA methylation. It usually occurs in repeated transposable DNA elements and is associated with genomic instability [10]. Studies have reported that hypomethylation of the MYC and RAS promoter regions can lead to the activation of proto-oncogenes [11]; hypomethylation of the IGF2 promoter region can lead to the loss of genetic imprinting [12]. DNA methylation is not limited to its expression level. Some methylation will bring about local distortion and shift, causing certain mutations. Studies have reported that the guanine-N7 methylation changes the hydrogen bonding mode of guanine and affects the stability of double-stranded DNA [13]. The chemical modification of DNA by endogenous and exogenous methylating agents (such as S-adenosylmethionine and N-methyl-N-nitrosourea) will produce a variety of genotoxic damage, of which N7- Methyl-2'-deoxyguanosine (m7dG) accounts for approximately 70-80% of total methylated lesions. The N7 methylation of dG does not promote mutant replication, and the polβ catalytic reaction across m7dG is slow but highly accurate [14]. In PDAC, previous studies confirmed the significance of DNA methylation in prognosis evaluation. Thus, constructing a DNA methylation model to predict PDAC prognosis for treatment optimization is worthwhile.

In this study, we analyzed the genome-wide methylation profiles of 184 cancer tissues from patients with PDAC in The Cancer Genome Atlas (TCGA) database. We established a methylation signature to assess patient prognosis Univariable Cox regression and Lasso regression. Using the Kaplan-Meier method and Receiver operating characteristic curves, we evaluated the diagnostic efficacy of the model and evaluated its clinical utility. The feasibility of the methylation model was further verified by validation dataset. Conclusively, we modeled a novel methylation signature predicting the inferior outcome of patients with PDAC.

## RESULTS

### Clinical characteristics of patients with PDAC

All 184 patients in this study were clinically and pathologically diagnosed with PDAC. The median age and median survival time of these patients was 65 years (range, 35–88 years) and 467 days, respectively. The 1- and 3-year OS rate of all patients was 64.86% and 11.35%, respectively. According to the standard 8^th^ AJCC TNM staging of pancreatic cancer, patients with PDAC included in our study were divided into stages I, II, III, and IV [15]. Simultaneously, we classified these patients into G1, G2, G3, and G4 in terms of histological grade based on the WHO classification. We obtained anatomical tumor subdivisions from different locations, including the pancreatic body, head, and tail. Table 1 summarizes the clinicopathological characteristics of the patients.

**Table 1:** Clinicopathological characteristics of PDAC patients from TCGA.

**Characteristics**	**Groups**	**Patients**					
		**Total(N=184)**		**Training dataset(N=129)**		**Validation dataset(N=55)**	
		**No.**	**%**	**No.**	**%**	**No.**	**%**
Gender	Male	102	55.43	71	55.04	31	56.36
	Female	82	44.57	58	44.96	24	43.64
Age at diagnosis	Median	65		65		66	
	Range	35-88		35-88		39-85	
	<65	84	45.65	60	46.51	24	43.64
	≥65	100	54.35	69	53.49	31	56.36
Pathological stage	I	21	11.41	11	8.53	10	18.18
	II	151	82.07	110	85.27	41	74.55
	III	4	2.17	3	2.33	1	1.82
	IV	5	2.72	3	2.33	2	3.64
	Unknown	3	1.63	2	1.55	1	1.82
Neoplasm histologic grade	Gx	2	1.09	1	0.78	1	1.82
	G1	32	17.39	21	16.28	11	20
	G2	97	52.72	70	54.26	27	49.09
	G3	51	27.72	36	27.91	15	27.27
	G4	2	1.09	1	0.78	1	1.82
Maximum tumor dimension	≤2cm	12	6.52	6	4.65	6	10.91
	>2cm	158	85.87	113	87.60	45	81.82
	Unknown	14	7.61	10	7.75	4	7.27
Anatomic neoplasm subdivision	Head of pancreas	145	78.80	106	82.17	39	70.91
	Body of pancreas	14	7.61	10	7.75	4	7.27
	Tail of pancreas	14	7.61	9	6.98	5	9.09
	Other	11	5.98	4	3.10	7	12.73
Lymph node metastasis	0	49	26.63	30	23.26	19	34.55
	1-3	76	41.30	58	44.96	18	32.73
	≥4	55	29.89	39	30.23	16	29.09
	unknown	4	2.17	2	1.55	2	3.64

### Identification of DNA methylation genes associated with the OS of patients in the training dataset

Using methylation level as a variable in the training dataset, we performed a univariate Cox proportional hazards regression analysis to identify DNA methylation markers related to OS in patients with PDAC. The results showed that a total of 646 DNA methylation gene loci were significantly correlated with PDAC OS (*P*<0.05). Subsequently, we used Lasso regression on methylated loci to refine these genes. Finally, based on the Lasso regression parameters lambda.min 0.06973033 and lambda.1se 0.2032676, we established a hazard ratio model consisted of four methylated genes, *CCNT1*, *ITGB3*, *SDS*, and *HMOX2* (Figure 1A, 1B). The risk score formulas of these genes were obtained as follows: risk score = −0.884 * methylation level of CCNT1 −1.934 * methylation level of ITGB3 −3.871 * methylation level of SDS −2.446 * methylation level of HMOX2. The prediction models of the relative gene expression levels of the four genes in the training and validation datasets were presented in the form of a heatmap (Figure 2A, 2B). In general, the methylated gene model obtained from the datasets of two different samples were the same and were related to prognosis, indicating that this model is meaningful. The differential expression of the four genes between tumor tissue and normal tissue was further verified by GEPIA (gene expression profiling interactive analysis) (http://gepia.cancer-pku.cn/detail.php), of which 179 were tumors and 171 were normal tissues. The results showed that these four genes (*CCNT1*, *ITGB3*, *SDS*, and *HMOX2*) were significantly overexpressed in PDAC tissues, suggesting that they may be potential biomarkers in patients with PDAC (Figure 3).

**Figure 1:** **LASSO regression analysis to construct PDAC specific diagnosis model.** (**A**) Least absolute shrinkage and selection operator (LASSO) coefficient profiles of differential methylation site. (**B**) Cross-validation for tuning parameter selection in the LASSO model, the two dotted vertical lines are drawn at the optimal values by lambda. min 0.06973033 and lambda.1se 0.2032676.

**Figure 2:** **Predicted DNA methylation marker heat map of PDAC patients based on risk scores tested in the training cohort and validation cohort.** (**A**) In the training data set, the relative gene expression level of the four DNA methylation genes in the prediction model based on the risk score is displayed in the form of a heat map. Each column represents a single patient in the combined verification cohort, ranked according to the predictor score, with the lowest score. Each row represents a gene in the model, sorted by gene's contribution to the score. Blue represents low risk, red represents high risk. (**B**) Same as above, perform the same operation in the verification data set for verification.

**Figure 3:** **The expression levels of four methylated genes in PDAC and normal tissues in TCGA database and their relationship with overall survival.** *, P<0.05.

### Association between four-DNA methylation signature and patient OS in the training and validation datasets

Kaplan-Meier analysis was performed on the training and validation datasets to determine the potential predictive value of this four-DNA methylation marker in prognosis. Using the median prognostic risk score as the cutoff point, each patient was assigned four DNA methylation markers in the high-risk (n=56) or low-risk (n=73) group of the training dataset. The average OS of the high-risk and low-risk groups was 13.1 months and 67.9 months, respectively. Patients in the high-risk group had a significantly worse prognosis than those in the low-risk group (*P*<0.0001) (Figure 4A). Similar results were observed in the validation dataset (Figure 4B). The risk scores in the training and validation datasets are shown in Figure 5A, 5B. Assign values according to the expression values of the selected four methylation genes, and then each patient specimen will get a total score. Finally, the patients were divided into high-risk group and low-risk group according to the total score. These results indicated that the new four-DNA methylation marker could distinguish high-risk patients from low-risk patients, which means that their prognosis in PDAC was predicted.

**Figure 4:** **Kaplan-Meier estimates "progression-free survival" because the diagnosis and progression of the diagnosis are predicted based on the 4-gene signature scores of patients in the training and validation cohort.** (**A**) In the training data set, high-risk patients have poor prognosis and short survival time, P<0.001. (**B**) The same is true in the validation data set, P=0.00018.

**Figure 5:** **Risk scores in training and validation datasets.** (**A**) The training dataset, (**B**) The validation dataset.

### Performance evaluation of the model established by four methylated genes

The AUC value is the area covered by the ROC curve. The larger the AUC, the higher the overall diagnostic efficiency. The four-DNA methylation marker had an AUC of 0.721 for 1-year OS and an AUC of 0.837 for 3-year OS (Figure 6A, 6B), indicating that the four DNA methylation markers have high sensitivity and specificity. Therefore, it could be used to predict the prognosis survival rate of patients with PDAC with high precision, which may be of great significance in clinical application.

**Figure 6:** **ROC curve shows sensitivity and specificity of four DNA methylation signature.** (**A**) The AUC of the 1-year OS of the four DNA methylation markers is 0.721. (**B**) The AUC of the 3-year OS of the four DNA methylation markers is 0.837.

### Differences in gene mutations in databases according to patient stratification by the model

Therefore, we divided all pancreatic cancer cases in TCGA database into high-risk and low-risk groups, and analyzed the differences in genetic mutations between the two groups (Figure 7). This revealed that the mutation rate of *TGFBR2* was 9% in the high-risk group and 1% in the low-risk group. The mutation rate of *SMAD4* was 32% in the high-risk group and 16% in the low-risk group. In addition, the enrichment analysis of these mutated genes in high-risk populations and other populations shows that there are differences in TGFBR2 and SMAD4 gene mutations between these two groups of patients (Figure 8). Further analysis showed that the potential drugs used between the two groups of patients were also different (Figure 9A, 9B), which can provide recommendations for clinical medication. For example, low-risk patients of SMAD4 gene mutation can be treated with transcription factor complex, histone modification, transcription factor binding, and high-risk patients can also use clinically actionable on this basis. By analyzing the abovementioned mutated genes and the survival time of patients, it can be concluded that the higher the mutation rate of *KRAS*, *CDKN2A*, and *TP53*, the shorter the survival time of patients, with statistical significance (Figure 10). Therefore, we can choose different treatment methods according to different populations to reduce the negative effects of excessive drug treatment.

**Figure 7:** **Differences in gene mutations between high-risk and low-risk PDAC patients.** One row represents a gene, and the top 15 is intercepted from it; One column is a sample, high risk group (n=78), low risk group (n=95). Different colors represent different types of mutations.

**Figure 8:** **Enriching mutant genes in high-risk groups and other groups, red represents high risk, gray represents ret.**

**Figure 9:** **Differences in the types of drugs used between high-risk patients and low-risk patients.** (**A**) The. high-risk patients, (**B**) The low-risk patients.

**Figure 10:** **Relationship between survival of PDAC patients and top six mutant driver genes.** (**A**) KRAS mutation, (**B**) SMAD4 mutation, (**C**) TGFBR2 mutation, (**D**) TP53 mutation, (**E**) BTBD11 mutation, (**F**) CDKN2A mutation)

### Comparison of the four-DNA methylation signature with other known prognostic biomarkers

Our results revealed that our new model is related to the prognosis of PDAC. To understand its clinical value, we compared the differences between the prognostic features of PDAC and previous studies. For example, the combination of *SRPX2* and *RAB31* may be an important prognostic marker for pancreatic cancer, with a 3-year AUC value of 0.748 [16]. Five critical lncRNAs are potential biomarkers for predicting the survival of patients with PDAC, with a 3-year AUC value of 0.742 [17]. The three hypomethylated genes are related to the differences in OS of pancreatic cancer patients, and the 3-year AUC value is 0.69 [18]. The ROC analysis of these biomarkers is the same as our analysis of the four DNA methylation markers. The results showed that the four DNA methylation markers are superior to other known prognostic biomarkers, including mRNAs, lncRNAs, and DNA alpha base type. These results are encouraging in showing that the four-DNA methylation model has better stability and reliability in predicting the OS of patients with PDAC.

## DISCUSSION

Owing to its molecular heterogeneity, PDAC remains one of the most invasive and fatal cancers worldwide. In the past, researchers have provided new insights into the molecular mechanism of PDAC and are committed to studying genetic differences. Recently, epigenetic regulation was also shown to have an indispensable role in PDAC. Increasing evidence demonstrated that DNA methylation is closely related to the biogenesis and prognosis of a variety of tumor types. For example, the DNA methylation patterns of *UBAC2* and *ELOVL2*, which are highly correlated with Chromosomal instability, provide potential prognostic value in Papillary thyroid carcinoma [19]. Hypermethylation of the *RASSF1A* and *BRCA1* promoters in circulating acellular tumor DNA is a biomarker for ovarian cancer [20]. *SARDH* methylation is an important prognostic factor for relapse-free survival in patients with RCC and has nothing to do with clinical prognosis, grade, stage, and metastatic status [21]. However, many of these studies are limited by small sample sizes or lack of validation as independent prognostic biomarkers.

In recent years, studies have shown that DNA methylation can be used as a biomarker for the early prediction and diagnosis of PDAC. Experimental evidence shows that the methylation status of *PCDH10* can predict the prognosis of patients with PDAC and has a significant effect on progression-free survival. High levels of *PCDH10* promoter methylation may help to identify patients at high risk of disease progression and more accurately stratify patients with PDAC for personalized clinical management [22]. Patients with hypomethylated *MUC1* and *MUC4* have lower OS and thus these are potential prognostic biomarkers of PDAC [23]. Hypomethylation of the *SERPINB5* promoter distinguishes PDAC from pancreatitis [24]. Because the tumor heterogeneity of PDAC is elevated, the mortality rate is very high, and thus prolonging the survival of patients is the focus of PDAC. Therefore, to reduce the mortality and improve the prognosis of PDAC, a molecular marker for the early screening of pancreatic cancer is urgently required. In this study, a novel four-gene pancreatic cancer prognostication model was constructed based on pancreatic cancer DNA methylation data and biological statistical methods. Single-factor and multi-factor Cox analysis was performed to further verify these methylation sites and their predictive value in the prognosis of PDAC. Finally, we confirmed a four-DNA methylation model consisting of *CCNT1*, *ITGB3*, *SDS*, and *HMOX2* by validating it as an independent prognostic indicator for patients with PDAC. The AUC of the ROC curves of the four-DNA methylation model in predicting 1-year survival was 0.721, while that predicting 3-year survival was 0.837. Therefore, these four markers have a good effect on the survival prediction of patients with pancreatic cancer.

Researchers have discovered that the four methylated gene loci identified in this study may have a crucial role in the development of cancer. Some researchers found that *CCND1* is regulated by EDG1 and has a new interaction function with estrogen receptor alpha (ERalpha), which is considered to have an important role in breast tumorigenesis [25]. Inhibition of ITGB3 expression can upregulate *miR-124-3p* and downregulate the expression of *lncRNA-H19*, thereby inhibiting the proliferation and invasion of ectopic endometrial cells and providing a new target for the treatment of endometriosis [26]. Inhibiting the expression of ITGB3 can increase the expression of *miR-124-3p* and thus inhibit the migration and invasion of gastric cancer, suggesting that *miR-124-3p* and ITGB3 may also be promising therapeutic targets for gastric cancer [27]. *HMOX2* may be related to the prognosis of patients with bladder cancer [28]. The G-888C polymorphism of the *SDS* (also known as *SDH*) gene may be related to the occurrence of diabetic retinopathy and has nothing to do with its progress. Its effect may be enhanced by interactions with the C-1214G polymorphism, but this weak association requires further study [29].

Cancer is closely related to genetic mutations. Although gene mutations are not enough to become a necessary condition for cancer development, the process of cancer is the common result of gene mutations, epigenetic regulation, and external factors [30]. Next-generation sequencing analysis of 50 cancer-related gene mutations, including driver genes in PDAC, found that the combination of *KRAS* and *SMAD4* mutations is an independent adverse prognostic factor in PDAC [31]. Several researchers identified a rare genetic mutation during a study of a group of cancer-prone families that may significantly increase the risk of individuals suffering from pancreatic cancer and other cancers in their lifetime. Identifying this previously unknown mutation may help researchers to routinely test individuals with a strong family history of pancreatic cancer to determine whether they carry a mutation in the relevant gene, *RABL3*. If confirmed, researchers may screen patients at an early stage of the disease [32]. In PDAC, *KRAS* gene mutations are closely related to its development [33]. Thus, we speculated whether patients with PDAC stratified according to the methylation model established in this study had genetic mutation differences. Obviously, the mutation rates of KRAS, TP53, and SMAD4 are higher in the high-risk group, and there are differences in the lower-risk group of TGFBR2 and SMAD4 mutations.

Although the functional mechanism of these four genes requires further study, the degree of methylation has a significant correlation with the prognosis of patients with PDAC and can be used as a potential therapeutic target for PDAC, thereby optimizing the treatment plan and prolonging the survival time of patients.

## CONCLUSIONS

In summary, through genome-wide analysis of the DNA methylation data of 184 patients with PDAC in TCGA database, we found that four hypomethylated genes were significantly associated with the poor prognosis of patients. We further demonstrated that the model has good accuracy and high feasibility, showing its potential as a new independent prognostic indicator and as an important tool to guide the clinical treatment of PDAC to improve patient prognosis prediction and management. Therefore, the results of this study are expected to provide new ideas for improving the clinical management of patients with PDAC.

## MATERIALS AND METHODS

### DNA methylation data of PDAC tissues from TCGA dataset

DNA methylation data and clinical information of patients were downloaded from TCGA PDAC subset by Illumina Human Methylation 450 Bead Chip. Only the data with patients’ survival data were selected for the subsequent analyses. Then, we studied the correlation between DNA methylation level and PDAC survival. A total of 184 samples containing 646 DNA methylation sites were finally included in this study. Based on the TCGA serial number, these 184 specimens were randomly divided into training (129 cases) and internal verification (55 cases) datasets. The training set aimed to identify and construct prognostic biomarkers, and the validation data set was used to verify the accuracy of these biomarkers in clinical predictive value.

### Statistical analyses

All statistical analyses were performed using the R statistical software package (R version 3.4.3) (https://cran.r-project.org/bin/windows/base/old/3.4.3/). Overall survival (OS) was defined as the time from the start of randomization to death from any cause. One-way Cox proportional hazard model analysis of the training dataset identified several significant methylation genes as candidate markers correlated with PDAC prognosis. Lasso regression analysis refined these genes and a four-gene model based on the Lasso regression parameters lambda. min 0.06973033 and lambda.1se 0.2032676, respectively, was generated. The ROC was obtained by plotting the true positive rate and the negative rate, which can reflect the relationship between sensitivity and specificity. The horizontal axis of the ROC curve represents the false positive rate, and the vertical axis represents the true positive rate. The area under the ROC curve was calculated for the performance of the methylation model, which could be utilized to build risk score formulas to predict the survival time of patients with PDAC. Patients were stratified into low-risk and high-risk groups according to the median risk score as the cut-off point. The Kaplan-Meier estimator with a log-rank test (Mantel-Cox) was used to calculate the cumulative survival time and compare the differences in OS between the two groups. The Kaplan-Meier curve was drawn by the Survival package, and the "pROC" package was utilized for the ROC analysis [34] (categorical variables of 1- and 3-year OS to compare against methylated biomarkers). The larger the AUC, the higher the risk of inferiority of the prognosis prediction of the PDAC methylation model. Additionally, the Maftools Bioconductor software package of R was used to analyze the somatic mutations of PDAC, and the mutation data were downloaded from TCGA and saved in the MAF file.
